The article "Blue Light Induces Down-Regulation of Aquaporin 1, 3, and 9 in Human Keratinocytes" was retracted in 2019. Reasons: manipulated images; unreliable results or conclusions; concerns about the data.

# Blue Light Induces Down-Regulation of Aquaporin 1, 3, and 9 in Human Keratinocytes

**DOI:** 10.3390/cells7110197

**Published:** 2018-11-03

**Authors:** Rosanna Avola, Adriana Carol Eleonora Graziano, Giovanna Pannuzzo, Venera Cardile

**Affiliations:** Department of Biomedical and Biotechnological Science, Section of Physiology, University of Catania, Via Santa Sofia, 97-95123 Catania, Italy; rosanna.avola@unict.it (R.A.); acegraz@unict.it (A.C.E.G.); giovanna.pannuzzo74@gmail.com (G.P.)

**Keywords:** aquaporin, blue light, photo aging, oxidative stress, keratinocytes, skin

## Abstract

The development in digital screen technology has exponentially increased in the last decades, and many of today’s electronic devices use light-emitting diode (LED) technology producing very strong blue light (BL) waves. Long-term exposure at LED-BL seems to have an implication in the dehydration of the epidermis, in the alterations of shape and number of the keratinocytes, and in the aging of the skin. Aquaporins (AQPs) are water membrane channels that permeate both water and glycerol and play an important role in the hydration of epidermis, as well as in proliferation and differentiation of keratinocytes. Thus, we have hypothesized that AQPs could be involved in the aging of the skin exposed to LED-BL. Therefore, we have examined the expression of AQPs in human keratinocytes exposed to LED-BL at dose of 45 J/cm^2^, used as an in vitro model to produce the general features of photo aging of the skin. The aim was to verify if LED-BL induces changes of the basal levels of AQPs. The keratinocytes exposure to LED-BL produced an increase of reactive oxygen species (ROS), an activation of 8-hydroxy-2’-deoxyguanosine (8-OHdG), an alteration of proliferating cell nuclear antigen (PCNA), and a down-regulation of AQP1, 3 and 9. These findings are preliminary evidences that may be used as starting points for further investigations about the mechanistic involvement of AQP1, 3, and 9 in LED-BL-induced skin aging.

## 1. Introduction

According to recent studies, 60% of people make a daily use of a digital device for about 6 h. Cell phones, computers, tablets, and flat-screen televisions are just among a few of the devices that use light-emitting diode (LED) backlight technology useful to improve the screen brightness and clarity. Thus, all people are globally exposed to different sources of blue light (BL) and for several hours a day. Previously, several studies focused on sight, memory, and sleep; more recently, interest has shifted towards skin aging because it has been shown that long-term exposure to LED-BL radiation disturbs the skin’s normal structure causing problems including its premature aging [1,2]. It was reported that a high exposure to LED-BL could accelerate signs of aging, increasing wrinkles, fine lines, dehydration, and hyperpigmentation generally associated with too much sun. Excessive LED-BL exacerbates the oxidation process, which turns in inflammation and alteration of skin barrier, making it more vulnerable to signs of aging [1,2,3,4]. Moreover, increased exposure to LED-BL results in a massive degradation of extracellular matrix (ECM) proteins such as collagen and elastin, produced by imbalance in equilibrium between the accumulation and degradation of ECM components that provide structural and functional support to the skin tissue. These ECM alteration turns in an increased activation of metalloproteases (MMP)-1, which induce overproduction of reactive oxygen species (ROS) such as singlet oxygen (^1^O_2_), superoxide anion (O^2−^), hydrogen peroxide (H_2_O_2_), hydroxyl radicals (OH^.^), formation of lipid hydroperoxides, protein carbonyls, 8-hydroxydeoxyguanosine (8-OHdG), and proliferating cell nuclear antigen (PCNA) and damage to the keratinocytes [5,6,7].

It is common that the cutaneous permeability barrier is essential for terrestrial life. A mixture of ceramides, sterols, and free fatty acids mediates the permeability barrier arranged as extracellular lamellar bilayers in the stratum corneum where there is a high presence of keratinocytes [8]. Although these studies indicate that this complex mixture of non-polar lipids is required for barrier homeostasis, little is known regarding the requirement for aquaporins (AQPs).

AQPs are expressed in various plants and microbes, including bacteria and yeast. A large number of plant aquaporins have been identified, called PIPs (plasma membrane intrinsic proteins) and TIPs (tonoplast intrinsic proteins) for their cellular expression patterns. In humans, AQPs are a family of membrane channels that comprises 13 homologous proteins regulated by factors that affect channel permeability or subcellular localization facilitating the transport of water and/or small solutes in response to changing of osmotic gradients. Functionally, AQPs can be divided into three different sub-family. AQP0, 1, 2, 4, 5, and 8 are water channels; AQP3, 7, 9, and 10, called aquaglyceroporins, transport water and other small solutes (e.g., glycerol and urea); AQP6, 11, and 12, unorthodox aquaporins, show a different sequence homology and are found in intracellular structures [9,10]. AQPs were identified in the major systems of the human body such as nervous, renal, cardiovascular, respiratory, reproductive, digestive, musculoskeletal, and integumentary [11]. An extensive set of studies examined the physiological and pathological role of AQPs in fluid absorption and secretion, cell signaling transduction, cell metabolism, cell migration, cell proliferation [12,13,14], stem cell differentiation [15,16], and primary or secondary neurodegeneration with the concomitance of different degree of inflammation [17,18]. In the skin, AQPs permit rapid, regulated, and selective water permeability playing a role in skin hydration, cell proliferation, migration, immunity, and wound healing [19]. Despite six skin AQPs have been identified (AQP1, 3, 5, 7, 9, 10) [20], the information on their expression in human skin is still strictly limited and highly controversial. In fact, although AQP1 and AQP3 presence in rat skin has been reported [20], AQP1 in human seems to be expressed in melanocytes and in vascular endothelial cells, where it facilitates water exchange between blood and skin. AQP7, found in adipocytes of skin dermis/hypodermis, is believed to be involved in glycerol transport [21,22]. AQP3, the most abundant skin aquaglyceroporin is able to enhancing keratinocytes proliferation and differentiation [23]. However, little is known about other, homologous AQPs. For example, much of the information about the localization and role of AQP9 remains unclear. Furthermore, actually, the most part of data about skin AQPs derives from research applied on rat and mouse models, and only a small number on human cellular systems.

Since keratinocytes, constituting 90% of the cells in the outermost layer of the skin, are the predominant cell type in the epidermis, the first aim of the present research was to confirm the damage induced by LED-BL exposure on human normal keratinocytes NCTC 2544 determining ROS formation, 8-OHdG expression, and PCNA activation. It was demonstrated that ROS reacting with DNA lead to DNA cleavage, and to endogenous DNA adducts formation, such as 8-OHdG, considered as an important biomarker of DNA damage. DNA damage and repair are also linked to the activation of PCNA, a nuclear protein marker of polymerase δ- (and/or ε-) dependent DNA synthesis. PCNA is directly involved in the major mechanism which eukaryote cells can remove bases from DNA that have been modified by various factor such as spontaneous hydrolysis or oxidation.

The second purpose was to determine the presence and behavior of some AQPs already identified in human skin and, in particular, AQP1, 3 and 9 in human keratinocytes NCTC 2544 exposed to 45 J/cm^2^ of LED-BL radiation.

The final purpose was to try to clarify the relationship between AQPs and skin aging induced by LED-BL arising from electronic devices.

## 2. Materials and Methods

### 2.1. Cell Culture

The human keratinocytes NCTC 2544 (provided by Interlab Cell Line Collection, Genoa, Italy), without HeLa cross-contamination, were cultured in Minimum Essential Medium (MEM) (Sigma-Aldrich, Milan, Italy) enriched with 10% heat-inactivated fetal bovine serum, (FBS, Sigma-Aldrich, Milan, Italy), 100 U/mL penicillin, 10 μg/mL streptomycin and 1% L-glutamine (Sigma-Aldrich, Milan, Italy) and incubated at 37 °C with 5% CO_2_ atmosphere. The medium was changed every 2–3 days.

### 2.2. Cell Treatment

NCTC 2544 cells were maintained in MEM growth medium up to a confluence of 40%–60%. A day before the experiments, the cell cultures was detached enzymatically (0.25% trypsin-0.02% EDTA), counted, and, in order to prevent cross irradiation, seeded in MEM medium with the maximum possible distance in 96 (1.5 × 10^3^), 24 (5 × 10^4^) or 6-well plates (3.0 × 10^5^). Twenty four hours after, the culture medium was discarded, and cells were washed with phosphate-buffered saline (PBS), and irradiated with 45 J/cm^2^ for 1.5 h at room temperature at wavelength below λ = 450 nm by LED-BL lamps in a Rayonet^®^ photochemical reactor (Southern New England Ultraviolet Company, Branford, CT, USA). To establish the quantity of radiation to use for the experiments and the IC_50_ value, at first, the keratinocytes were irradiated with 5, 10, 15, 25, 45, 50, or 85 J/cm^2^ and evaluated for cell viability. Immediately after irradiation, the cultures replaced by fresh medium were incubated in a controlled humidified cell culture incubator (37 °C, 5% CO_2_/95% air) and after 24 h used to check the effect of LED-BL on cell viability, oxidative stress, and some gene and protein parameters linked to photo damage. Additionally, NCTC 2544 cultures were visualized using a Zeiss phase contrast microscope (Nikon Instruments, Melville, NY, USA), equipped with an Olympus ALTRA 20 digital camera and AnalySIS getIT software (Olympus Soft Imaging Solutions, Münster, Germany) at the beginning and the end of every experiment and after medium changes.

### 2.3. Cell Viability

Cell viability was evaluated as previous described by Graziano et al. [24]. Cells were seeded at the density of 1.5 × 10^3^ cells/cm^2^ in 96-well plates and incubated at 37 °C, 5% CO_2_/95% air for 24 h with growth medium. Next, the culture medium was substituted with PBS and experimental cultures were irradiated. After irradiation, the keratinocytes were maintained in culture medium. Twenty four hours after, 200 μL of tetrazolium salt 3-(4,5-dimethylthiazol-2-yl)-2,5-diphenyltetrazolium bromide (MTT) (Sigma-Aldrich, Milan, Italy) in PBS at final concentration of 5 μg/mL were added into each well for 3 h at 37 °C. After, the supernatant was removed and replaced with 100 μL of dimethylsulphoxide (DMSO) to solubilize the blue formazan crystals. The absorbance at λ = 550 nm was measured by a microplate spectrophotometer reader (Titertek Multiskan, DAS, Milan, Italy). The data were averaged (three experiments in triplicate) and represented as percentage of viability with respect to untreated controls.

### 2.4. Determination of ROS

The level of intracellular ROS was assessed by measuring the oxidation of 2′,7′-dichlorodihydrofluorescein diacetate (H2-DCFDA) (Sigma-Aldrich, Milan, Italy). H2-DCFDA diffuses through the cell membrane and is enzymatically hydrolyzed by intracellular esterase to the non-fluorescent H2-DCF [25]. Intracellular ROS are able to oxidize H2-DCFDA to the fluorescent 2′-7′-dichlorofluorescein (DCF), whose intensity of fluorescence is directly proportional to the levels of intracellular ROS. Briefly, 5 mM of H2-DCFDA were added to the keratinocytes cultures. The cells were kept in a humidified atmosphere (5% CO_2_, 37 °C) for 10 min and then washed in PBS. Fluorescence was measured at excitation/emission wavelengths of λ = 480/535 nm using a Hitachi F-2000 spectrofluorimeter (Hitachi, Tokyo, Japan). Values (three experiments in triplicate) were expressed as relative fluorescence units normalized versus the level of ROS in the control cells.

### 2.5. Determination of 8-Hydroxy-2’-Deoxyguanosine (8-OHdG)

The amount of DNA damaged was analyzed by the quantification of 8-OHdG production. NCTC 2544 cells (5 × 10^4^) were seeded on 24-well plates and exposed to 45 J/cm^2^ LED-BL radiation. After 24 h, the cells were fixed with 4% paraformaldehyde in PBS at 4 °C for 2 h. Next, the cells were incubated with 0.05 N HCl for 5 min on ice, washed with PBS and incubated with 300 μL of RNAse (100 μg/mL dissolved in 150 mM NaCl and 15 mM sodium citrate) for 1 h at 37 °C. Subsequently, NCTC 2544 were dehydrated in a graded alcohol series (35, 50, and 75% ethanol), washed in PBS and incubated with 300 μL of 0.15 M NaOH in 70% ethanol for 4 min to denature DNA in situ. The alkaline solution was neutralized by 70% ethanol containing 4% formaldehyde. After, the cells were treated with 50%, 35% ethanol, and PBS. Next, 300 μL of proteinase K (5 μg/mL in 20 mM Tris and 1 mM EDTA, pH 7.5) were added to the cells and incubated for 10 min at 37 °C. To prevent non-specific binding the samples were blocked with 5% BSA for 1 h at room temperature. The cells were subsequently incubated overnight at 4 °C with a primary antibody direct against anti-8-OHdG (sc-393870; Santa Cruz Biotechnology, Santa Cruz, CA, USA; 1:200 dilution). The following day, cells were washed with PBS and incubated for 1 h at room temperature with a fluorescein isothiocyanate conjugated goat anti-mouse (12-506, FITC; Millipore, Milan, Italy; 1:400 dilution) antibody. After washed with PBS the level of binding was measured at excitation/emission wavelengths of λ = 488/519 nm using a Hitachi F-2000 spectrofluorimeter (Hitachi, Tokyo, Japan). The cell density was assessed by the incubation of all experimental cultures with DAPI (Invitrogen, Milan, Italy; 1:10000 dilution) for 10 min at room temperature and the measure of fluorescence intensity (λ = 346/460 nm). Values (three experiments in triplicate) were expressed as fold change versus untreated control.

### 2.6. RT-PCR

The reverse transcriptase-polymerase chain reaction RT-PCR assay was performed and analyzed as previously described in Avola et al. [18]. The complementary DNA cDNAs were synthesized from the total RNA samples by using the QuantiTect Reverse Transcription Kit (Qiagen, Milan, Italy) according to the manufacturer’s protocol. Aliquots of cDNA were amplified using the following specific primers sequences:

**AQP1**: 5’-CTCTCTGTAGCCCTTGGACACCTC-3’ (Forward),

    5’-GGCATCCAGGTCATACTCCTCCAC-3’ (Reverse);

**AQP3**: 5′-ACCTTTGCCATGTGCTTCCT-3’ (Forward),

    5′-CTGGCACCCAGCACAATG-3’ (Reverse);

**AQP7**: 5′- CTGACTCCTGTTGTCCTCCACCTC-3’ (Forward),

    5′-AAATGGTCTCCTGGTCCGTGATAG-3’ (Reverse);

**AQP9**: 5′-GATACTCCTCATAATCGTCTTTGC-3’ (Forward),

    5′-AAGACTGAGTCAGGCTCTGGATGG-3’ (Reverse);

**AQP10**: 5′-ATAGCCATCTACGTGGGTGGTAAC-3′ (Forward),

    5′-TTTGTGTTGAGCAGACACCAGATC-3′ (Reverse);

**GAPDH**: 5’-TCAACAGCGACACCCAC-3’ (Forward),

    5’-GGGTCTCTCTCTTCCTCTTGTG-3’ (Reverse).

For PCR analysis, a concentration of 100 ng/reaction of template cDNA was added to the reaction mix containing 1x Rotor-Gene SYBR Green PCR Master Mix (Qiagen, Milan, Italy), 1 μM of each primer (forward and reverse) and RNase-free water to a final reaction volume of 25 μL. PCR was performed using the following program: initial activation step 95 °C 10 min, denaturation 95 °C 10 s, annealing 60 °C 30 s, extension 72 °C 30 s (40 cycles), final extension 72 °C 10 min. RT-PCR was followed by melting curve analysis to confirm PCR specificity. Each reaction was repeated three times and threshold cycle average was used for data analysis by Rotor-gene Q software. Target genes were normalized against GAPDH. Amplification products were separated by electrophoresis in a 2% agarose gel in 0.045 M Tris–borate/1mM EDTA (TBE) buffer. Each amplification was carried out in duplicates in four different experiments. The 2^−ΔΔCT^ method was used to calculate the difference in CT value between the LED-BL-treated samples and untreated controls. Results were then normalized to an endogenous reference gene (GAPDH) whose expression is constant in all groups.

ΔΔCT = (CT Target − CT Reference gene)_treated_ − (CT Target − CT Reference gene)_untreated_

The results were reported as fold change of LED-BL-treated cells vs. untreated control.

### 2.7. Western Blot

Keratinocytes NCTC 2544 were lysed with buffer M-PER Mammalian Protein Extraction Reagent (Pierce, Fisher Scientific, Milan, Italy) and vortexed for 30 min on ice. The insoluble debris was removed by centrifugation at 15,000× *g* for 15 min at 4 °C [26]. The protein quantification was performed by the bicinchoninic acid assay (BCA assay; Pierce, Fisher Scientific, Milan, Italy). The proteins in equal amount (40 μg) were separated by 4–12% bolt gel (Invitrogen, Milan, Italy) and electrophoretically transferred to nitrocellulose membranes (Invitrogen, Milan, Italy) in a wet system (Invitrogen, Milan, Italy). The transfer of proteins was verified by staining the nitrocellulose membranes with Ponceau S. Membranes were blocked in Tris-buffered saline containing 0.01% Tween-20 (TBST) and 5% non-fat dry milk for 1 h at room temperature. Primary antibodies anti-AQP1 (sc-20810), anti-AQP3 (sc-518001), anti-AQP7 (sc-376407), anti-AQP9 (sc-28623) (all from Santa Cruz Biotechnology, DBA, Milan, Italy, 1:200 dilution), anti-AQP10 (AV50244, Sigma Aldrich, Milan, Italy; 1:200 dilution), and anti-PCNA protein expression (A300-277A-M; Bethyl Laboratories, Tema Ricerca, Bologna, Italy, 1:2000 dilution) were diluted in TBST and incubated on the membranes overnight at 4 °C. Blots were rinsed three times in PBS and the appropriate HRP-conjugated secondary antibody was incubated for 1 h at room temperature (goat anti-rabbit, 1:20000 dilution; goat anti-mouse, 1:5000 dilution, both Santa Cruz Biotechnology, DBA, Milan, Italy). Antibodies were detected with chemiluminescent solution (Pierce, Fisher Scientific, Milan, Italy) and visualized by Uvitec Alliance LD9 gel imaging system (Uvitec, Cambridge, UK). Bands were measured densitometrically and their relative density was calculated based on the density of the α-tubulin bands in each sample. Values of arbitrary densitometric units (A.D.U.) (three experiments in triplicate) corresponding to signal intensity were expressed as fold of change with respect to untreated control.

### 2.8. Statistical Analysis

The assays were performed at minimum three times in triplicate and the mean ± standard error of mean SEM for each value was calculated. Student’s t-test for paired and variance analysis (ANOVA) for unpaired data were used. All statistical analyses were made using the statistical software package SYSTAT, version 11 (Systat Inc., Evanston IL, USA). A value of *p* < 0.05 was considered to indicate a statistically significant difference.

## 3. Results

### 3.1. Cell Viability

Before to perform the experiments, we determined the IC50 value and so established what quantity of LED-BL energy to use for the several assays by exposing keratinocytes NCTC 2544 to 5, 10, 15, 25, 45, 50, or 85 J/cm^2^. After 24 h from irradiation, the MTT assay was performed. Compared to non-exposed control cells, the viability decreased in dose-dependent manner. Keratinocytes, in fact, irradiated with 5, 10, 15, 25, 45, 50, and 85 J/cm^2^ showed a viability of 95 ± 2, 81 ± 3, 72 ± 6, 53 ± 4, 42 ± 6, and 23 ± 4%, respectively (Figure 1), and a IC_50_ value of 47.8 ± 2. So, at 45 J/cm^2^ irradiation, the cell viability reduced by about 50%. Since viable cells with active metabolism convert MTT into purple formazan product, the sharp decline in formazan product due to irradiation with 45 J/cm^2^ indicates that this dose (corresponding almost to IC_50_) significantly impairs the mitochondrial metabolic activity. For this reason, we selected the 45 J/cm^2^ energy to assess the pathways involved in LED-BL aging.

### 3.2. Production of ROS

ROS have been reported to be involved in cell damage induced by light radiation. In order to characterize the level of oxidative stress and assess the changes of intracellular ROS caused by LED-BL irradiation, confluent NCTC 2544 were treated with H2-DCFDA. Twenty-four hours after treatment, the fluorescence signal, indicator of intracellular oxidants, was measured and compared to non-exposed control cells. H2-DCFDA can be taken up into cells, and then oxidized by ROS to its fluorescent derivative DCFDA [27]. Compared to non-exposed control cells, fluorescent DCFDA increased significantly in 45 J/cm^2^ LED-BL exposed cells (80 ± 15%) indicating a very strong ROS production (Figure 2).

### 3.3. Determination of Collagen Type I and DNA Damage

The relationship between LED-BL and damage in human keratinocytes was further demonstrated by the levels of 8-OHdG [28,29] and PCNA [30]. Compared to the controls, 8-OHdG fluorescence generated in LED-BL-treated cells was significantly higher (Figure 3A). Immunoblotting (Figure 3B) and immunofluorescence (Figure 3C) staining confirmed increased production of PCNA in human NCTC 2544 after exposure to LED-BL, while it was almost absent in untreated control cells (Figure 3B,C).

### 3.4. Determination of AQPs Expression Profile

In order to investigate the effect of LED-BL exposure on AQP1, 3, 7, 9, and 10 and try to find a link between LED-BL-induced damage and levels of expression of these channel proteins, we performed RT-PCR and Western blot in human keratinocytes NCTC 2544 untreated and treated with LED-BL radiation. The results showed that compared to each untreated control, LED-BL exposure induced very significant AQP1, 3 and 9 down-regulation (Figure 4). In particular, at the mRNA level the most decreased was AQP3, at the protein level it was AQP1. Finally, AQP7 and AQP10 were never detected at both mRNA and protein level.

## 4. Discussion

The results of our study confirmed that LED-BL at 45 J/cm^2^ damages human skin keratinocytes NCTC 2544 and demonstrated that it induces a down-regulation of cell membrane channel proteins AQP1, 3 and 9.

In our modern daily life, our skin is extensively exposed to artificial LED-BL that illuminates the screens of all electronic devices such as computers, televisions and cell phones. Although the energy emitted is weak, people tend to be very close to the light source and spend a very high quantity of hours in a day in front to digital devices, reaching a mean of 8.5 h of direct exposition, value destined to grow incessantly [31].

The premature skin aging is characterized by presence of wrinkles, sagging, pigmented spots, dryness, and loss of elasticity and resilient associated with deeper modifications of structure of the skin [32,33]. In particular, it is largely known that the modification of shape and number of keratinocytes and fibroblasts is linked to the up- or down-regulation of intra- and extracellular proteins via multifarious cell signaling pathways. Histopathological analysis revealed the massive deterioration of aged skin characterized by a breakdown of collagen type I and elastic fiber as a direct consequence of the activation of MMPs leading to the development of wrinkle formation [34,35,36,37]. Actually, despite a growing number of children and adults being increasingly exposed to LED-BL, their effects on skin and the rate of damage are poorly known.

In the last years, to study the influence and the biological effects of LED-BL, many researchers applied different LED-BL radiation conditions such as wavelength, dose, intensity, exposure time or light sources with different and sometimes broad spectra partly with ultraviolet radiation-A (UVA), so the achievement of a univocal result is complicated. As reported by Gilchrest [38], the observation that the aging of sun-exposed skin resembles to chronologic aging lead to the hypothesis that both are mediated by the same cause [39]. As it is known, ROS, that escape the cell defenses, are signaling molecules able to induce damage to DNA, accumulation of mitochondrial DNA mutations [40], and replicative senescence [41]. Overproduction of these ROS, in fact, may provoke oxidation of polyunsaturated fatty acids (PUFAs) in cellular membranes through free radical chain reactions and form lipid hydroperoxides as primary products. Among these lipid peroxidation products, 4-hydroxy-2-nonenals (4-HNE) represents one of the most bioactive and well-studied lipid alkenals. 4-HNE can modulate a number of signaling processes mainly through forming covalent adducts with nucleophilic functional groups in proteins, nucleic acids, and membrane lipids [42].

Recently, Rascalou et al. [31] demonstrated that the cell cultures exposure to 99 J/cm^2^ of blue light is equivalent to cells exposed to the screen of an electronic device for 1952 h in real life. Thus, in our in vitro system, we tried to obtain a model of LED-BL exposition treating NCTC 2544 with 5, 10, 15, 25, 45 50, and 85 J/cm^2^ [43]. The MTT results showed a dose-dependent reduction of viability and confirmed the dose of 45 J/cm^2^ inducing cell mortality near to 50% (IC_50_ value= 47.8 ± 2 %). In parallel, after irradiation, we observed morphological changes, because the keratinocytes seem to be rounded and shrunken (data not shown). Moreover, we demonstrated that ROS level was increased, as well as 8-OHdG and PCNA amount, these latter markers of DNA damage. There is extensive experimental evidence that oxidative damage permanently occurs to lipids of cellular membranes, proteins, and DNA. ROS can attack base and sugar moieties in DNA yielding a variety of lesions such as apurinic and apyrimidinic sites, DNA strand breaks, or oxidized bases. Apyrimidinic sites are one of the most common lesions in the cellular DNA, which can also be formed spontaneously, or by the action of DNA glycosylases on modified bases. In nuclear and mitochondrial DNA, 8-hydroxy-2’-deoxyguanosine (8-OHdG) or 8-oxo-7, 8-dihydro-2’-deoxyguanosine (8-oxodG) is one of the predominant forms of free radical-induced oxidative lesions, and has therefore been widely used as a biomarker for oxidative stress and carcinogenesis. Increased ROS levels are also associated with increases in mitogen-activated protein kinases (MAPK) activation and the expression of PCNA and cyclin D1, two of the most important modulators directly involved in cell proliferation and cell cycle progression. PCNA is a homotrimeric protein that forms a sliding clamp around DNA and acts as a processivity factor for the replicative polymerase. PCNA also interacts with many other proteins such as translesion synthesis polymerases, which plays a crucial role in targeting them to the damage site and stimulating their enzymatic activity. Hence, PCNA is an essential protein that functions in DNA replication, repair, recombination, damage tolerance, and cell cycle control. Its deregulation is an indication of cellular damage.

Since hydration remains one of the major approaches for prevention against skin photo aging and little it is known about the molecular mechanism of LED-BL induced skin dehydration [44], we hypothesized that in addition to the damage described above, LED-BL could induce a change in the expression of the aquaporins. In mammalian skin, several kinds of AQPs such as water channels and aquaglyceroporins have been identified; specifically, AQP1, 3, 5, 7, 9, and 10 are involved in maintenance of hydration state of skin barrier function, and for this reasons, are strictly related to skin physiology [12,13,45,46].

AQP3 was the first and the most abundant AQP detected in epidermis, and it is located in keratinocytes plasma membrane where it seems to have a role in the transport and metabolism of glycerol and, consequently, of water, to ensure a correct epidermis hydration [12,46,47]. Recently, in knockout mice has been shown that AQP3 has a functional role in the maintenance of skin hydration and consequently changes in the regulation of AQP3 may be the cause or consequence of skin dehydration [48]. In particular, AQP3 down-regulation is linked to skin glycerol content reduction, water holding capacity diminution, elasticity decline, hydration decrease, and wound healing delay [49,50]. Moreover, a relevant correlation between mechanical and biosynthetic defects and AQP3 down-regulation was found [51]. A reduction in glycerol content, in fact, results in an impaired epidermal proliferation [46] since glycerol is an important metabolite of skin cells, being involved in ATP production and in membrane lipids biosynthesis [52]. Mice deficient in AQP3 have dry skin with reduced stratum corneum hydration, decreased elasticity and impaired biosynthesis. Mechanistic analysis of the altered skin phenotype in AQP3 deficiency suggested that the glycerol rather than the water is important in skin physiology. The barrier function as well as the mechanical properties of the skin does not only depend on its water content, but more importantly, on the state and molecular organization of lipid and protein components. These properties can be affected by hydration and by the addition of other small polar molecules. For example, the presence of glycerol in hydrated model skin lipids in a liquid crystalline state impedes the transition into a crystalline state at dry conditions, as compared to the same lipid mixture in the absence of glycerol. These observations indicate that glycerol can maintain the physical properties of hydrated lipid systems under dry conditions [53]. Glycerol is also used in commercial skin care lotions and creams where the beneficial function of this compound is ascribed to its hygroscopic properties,

As regard AQP9, it was found in most part of keratinocytes granular layer where AQP3 expression was diminished [54]. Like AQP3, AQP9 is an aquaglyceroporin that plays a central role in glycerol metabolism, in cell motility and it could be an additional player in wound healing, but its function in skin has not yet been studied extensively. It was observed that in cultured human keratinocytes treated with high concentration of calcium as differentiating agent significantly the AQP9 expression increases, suggesting the possibility that AQP9 plays a role in highly differentiated keratinocytes [55].

More controversial appears the role of AQP1: AQP1 mRNA was shown in human melanocytes and, in smaller amounts, in epidermal cells. Despite the observation that water transport by AQP1 seems not to have a significant role in skin hydration, recent discoveries suggest that AQP1 is involved in the cell shape and migration [56], in the melanocytes growth, and in melanosome transfer to keratinocytes [20]. In any case, the knowledge of many features of different skin AQPs like AQP1, 9, and 10, including their function and expression, remains elusive.

For this reason, at the beginning of our study the purpose was to perform systematic analysis of all aquagliceroporins (AQP3, 7, 9, and 10) important for glycerol homeostasis that, as reported above, is an important metabolite of skin cells. Moreover, considering that in our precedent study, we have largely supposed a relevant role of AQP1 in the sustaining of the physiological homeostasis such as in the promotion of proliferation and differentiation in several cell systems [15,16], we have decided to detect also in our experimental conditions AQP1. The results demonstrated that in keratinocytes the 45 J/cm^2^ LED-BL radiation induces a general decrease in AQP1, 3, 9, while no presence of AQP7 and 10 was found in our experimental conditions.

To the best of our knowledge, this is the first study that analyzes the effects of LED-BL on AQPs expression. Some studies demonstrated that UV induces generation of ROS that activates MEK/ERK pathway leading to AQP3 down-regulation in cultured human skin keratinocytes [44]. Moreover, the pretreatment with antioxidant like chrysin exerts a protective effect against apoptosis, ROS overproduction, cyclooxygenase-2, (COX-2) induction and AQP3 down-regulation caused by UVA and ultraviolet radiation-B (UVB) radiation on keratinocytes cultures in a dose-dependent manner [57]. However, the detailed role of AQP1, 3 and 9 in LED-BL induced dry skin warrants further investigation.

Taken together, our results demonstrated that LED-BL exposure seems to be involved in premature skin aging. Moreover, in our experimental condition, keratinocytes react to LED-BL down-regulating AQP1, 3 and 9. These findings are preliminary evidences that may be used as starting points for further investigations about the mechanistic involvement of AQP1, 3, and 9 in LED-BL-induced skin aging. In any case, skin protection against artificial visible light should no longer be neglected.

## Figures and Tables

**Figure 1:** Cell viability assessed by MTT assay of keratinocytes NCTC 2544 treated with light-emitting diode blue light (LED-BL) at 5, 10, 15, 25, 45, 50, and 85 J/cm^2^. Each point represents mean ± SEM of three separate experiments performed in triplicate. * Significant versus untreated control, *p* ≤ 0.05.

**Figure 2:** Production of reactive oxygen species (ROS) measured by 2’, 7’dichlorodihydrofluorescein diacetate (H2-DCFDA) assay. The results reported as relative fluorescence unit showed a significantly increased ROS level after treatment of NCTC 2544 with LED-BL at 45 J/cm^2^. Data represent mean ± SEM of three separate experiments performed in triplicate. * Significant versus untreated control; *p* ≤ 0.05.

**Figure 3:** Determination (**A**) of 8-OHdG by immunofluorescence, and (**B**,**C**) of PCNA protein by Western blot in NCTC 2544 untreated or treated with LED-BL at 45 J/cm^2^. (**A**,**C**) protein expression calculated as fold change versus untreated control (Control); * significant versus untreated control; *p* ≤ 0.05.

**Figure 4:** Determination of aquaporin (AQP)1, 3, and 9 by (**A**, **B**, and **C**, respectively) RT-PCR and (**E**, **F**, and **G**) Western blot in NCTC 2544 untreated or treated with LED-BL at 45 J/cm^2^. Values reported in (**D**) for RT-PCR and (**H**) for Western blot, respectively, were expressed as fold change versus untreated control. * Significant versus untreated control; *p* < 0.05.
